# Dorsomorphin Promotes Survival and Germline Competence of Zebrafish Spermatogonial Stem Cells in Culture

**DOI:** 10.1371/journal.pone.0071332

**Published:** 2013-08-01

**Authors:** Ten-Tsao Wong, Paul Collodi

**Affiliations:** Department of Animal Sciences, Purdue University, West Lafayette, Indiana, United States of America; National University of Singapore, Singapore

## Abstract

Zebrafish spermatogonial cell cultures were established from *Tg(piwil1:neo);Tg(piwil1:DsRed)* transgenic fish using a zebrafish ovarian feeder cell line (OFC3) that was engineered to express zebrafish Lif, Fgf2 and Gdnf. Primary cultures, initiated from testes, were treated with G418 to eliminate the somatic cells and select for the *piwil1:neo* expressing spermatogonia. Addition of dorsomorphin, a Bmp type I receptor inhibitor, prolonged spermatogonial stem cell (SSC) survival in culture and enhanced germline transmission of the SSCs following transplantation into recipient larvae. In contrast, dorsomorphin inhibited the growth and survival of zebrafish female germline stem cells (FGSCs) in culture. In the presence of dorsomorphin, the spermatogonia continued to express the germ-cell markers *dazl*, *dnd*, *nanos3*, *vasa* and *piwil1* and the spermatogonial markers *plzf* and *sox17* for at least six weeks in culture. Transplantation experiments revealed that 6 week-old spermatogonial cell cultures maintained in the presence of dorsomorphin were able to successfully colonize the gonad in 18% of recipient larvae and produce functional gametes in the resulting adult chimeric fish. Germline transmission was not successful when the spermatogonia were cultured 6 weeks in the absence of dorsomorphin before transplantation. The results indicate that Bmp signaling is detrimental to SSCs but required for the survival of zebrafish FGSCs in culture. Manipulation of Bmp signaling could provide a strategy to optimize culture conditions of germline stem cells from other species.

## Introduction

The zebrafish embryo is an ideal model for in vivo analysis of germ cell determination and migration during early development [1], [2], however complementary in vitro studies of zebrafish germ cell growth and differentiation have been lacking due to the absence of suitable cell culture systems. Mouse spermatogonial stem cell (SSC) and female germline stem cell (FGSC) cultures have proven to be valuable in vitro models for studies of germ cell differentiation and been used for the production of transgenic and knockout mice [3], [4], [5], [6]. Recently, our lab used a drug selection strategy to establish zebrafish FGSC cultures that were initiated from *Tg(piwil1:neo);Tg(piwil1:DsRed)* transgenic fish. The *Tg(piwil1:neo);Tg(piwil1:DsRed)* fish express Neo and DsRed under the control of the *piwil1* promoter enabling the use of G418 selection to isolate the *piwil1:neo* expressing FGSCs. Using this method a homogeneous population of FGSCs were selected and maintained for more than 6 weeks in culture during which the cells continued to express multiple germ cell markers. Following transplantation into recipient larvae, the cultured FGSCs successfully colonized the gonad of the host and produced functional gametes in the adult chimeric fish [7].

Since *piwil1* is also expressed in the germ cell lineage of male zebrafish [8], [9], [10], in this paper, we apply the same drug selection strategy to establish zebrafish spermatogonial cell cultures from the gonad of male *Tg(piwil1:neo);Tg(piwil1:DsRed)* fish. Previous attempts to establish long-term spermatogonial cell cultures from zebrafish were ineffective due to spontaneous differentiation of the spermatogonia to non-proliferating spermatids [11], [12] and to the cultures becoming overgrown by testicular somatic cells [13]. To avoid these problems, primary cultures were initiated from the testes of *Tg(piwil1:neo);Tg(piwil1:DsRed)* fish and treated with G418 to select Neo-expressing spermatogonia and eliminate somatic cells. A key component of the culture system was the addition of dorsomorphin to block Bmp signaling which prevented the spontaneous differentiation of the zebrafish spermatogonia and prolonged their survival in culture. The action of dorsomorphin on spermatogonia in culture is consistent with results of previous studies showing that mutation of the Bmp type I receptor impairs germ cell differentiation in zebrafish testis [14] and the addition of exogenous BMP promotes mouse spermatogonial differentiation in culture [15], [16]. In our study, inhibition of Bmp signaling also enhanced the capacity of cultured spermatogonia to colonize the gonad following transplantation into recipient larvae and produce functional gametes in the adult chimeric fish.

## Materials and Methods

### Animals and Ethics

Zebrafish were maintained and staged as previously described [17]. All of the experimental procedures and protocols described in this study were approved by the Purdue University Animal Care and Use Committee and adhered to the National Research Council’s Guide for Care and Use of Laboratory Animals.

### Immunocytochemistry and Histology

Gonads dissected from zebrafish were fixed with either 4% paraformaldehyde in phosphate-buffered saline (PBS) or Bouin’s fixative at 4°C overnight, and then processed through successive treatments of ethanol (50%, 70%, 95%, and 100%) followed by two xylene baths and embedded in paraffin. The serial paraffin sections (5 µm) were prepared for immunocytochemical staining to visualize Neo and Vasa within the testicular tissues of *Tg(piwil1:neo)* [7] according to published protocols [18], [19]. Tissue sections were treated with mouse anti-neomycin phosphotransferase II monoclonal IgG (1∶500 dilution, Abcam) and rabbit anti-zebrafish Vasa antiserum [20] (1∶4000 dilution) and then stained with Alexa Fluor 488 AffiniPure goat anti-mouse IgG and Cy3 AffiniPure goat anti-rabbit IgG (1∶500 dilution, Jackson ImmunoResearch Lab, Inc.). Neo and Vasa expression was evaluated by examining the tissue sections by fluorescence microscopy using a Nikon Eclipse TE200 microscope (Nikon, Tokyo, Japan) equipped with a RT Slider digital camera (Spot Imaging Solution, Sterling Heights, MI, USA). The sections were stained with hematoxylin-eosin for histological examination by light microscopy.

### Spermatogonial Cell and FGSC Cultures

To initiate the spermatogonial cell cultures, testes dissected from 2- to 3-month-old *Tg(piwil1:neo);Tg(piwil1:DsRed)* transgenic fish [7] were minced and dissociated in collagenase solution (0.2% collagenase, Invitrogen and 0.002% DNase I, Sigma-Aldrich in PBS; 28.5°C, 1 hour). Using Percoll discontinuous gradient centrifugation, loach spermatogonia were found in the 30, 33 and 36% fractions [21]; zebrafish spermatogonia were found in the 25, 30, 33 and 36% fractions with the majority observed in 25 and 30% fractions (unpublished results). Hence, zebrafish spermatogonia were partially purified by passing the dissociated tissue through a discontinuous Percoll gradient (20–40%) and the resulting cell suspension was seeded into individual wells (cells from 1 to 1.5 fish/well) of a 12-well plate. Each of the wells was previously seeded with 2×10^5^ growth arrested feeder cells. The feeder cell lines used for this work OFC3, OFC3LF (transfected with zebrafish Lif and Fgf2) and OFC3LG (transfected with zebrafish Lif and Gdnf) were irradiated for 8 Krads as previously described [7]. Modified StemPro®-34 SFM culture medium (Invitrogen) supplemented with minimal essential medium (MEM) vitamin solution (Invitrogen), MEM nonessential amino acid solution (Invitrogen), 5% KnockOut™ serum replacement (Invitrogen), 0.4% BSA (Sigma-Aldrich), 10 µg/ml insulin (Sigma-Aldrich), 100 µg/ml transferrin (Sigma-Aldrich), 60 µM putrescine (Sigma-Aldrich), 30 nM sodium selenite (Sigma-Aldrich), 3 mg/ml D-(+)-glucose (Sigma-Aldrich), 1 µl/ml DL-lactic acid (Sigma-Aldrich), 2 mM l-glutamine (Sigma-Aldrich), 50 µM 2-mercaptoethanol (Sigma-Aldrich), 100 µM ascorbic acid (Sigma-Aldrich), 10 µg/ml d-biotin (Sigma-Aldrich), 30 ng/ml β-estradiol (Sigma-Aldrich), 60 ng/ml progesterone (Sigma-Aldrich), 2 µM retinol (Sigma-Aldrich), 40 ng/ml human epidermal growth factor (EGF) (StemGent, Cambridge, MA, USA), 1% FBS (Harlan), 1% fish serum (East Coast Biologics, Inc., North Berwick, ME, USA) and 30% conditioned medium [7], [22]. Dorsomorphin (Chemdea, Ridgewood, NJ, USA) was added to the medium at a final concentration of 0, 1, 2, 4, or 8 µM (in final 0.4% dimethyl sulfoxide, Sigma-Aldrich). The cells were maintained at 28.5°C in an atmosphere of 3% carbon dioxide and the medium was replaced every 3–4 days. Following G418 selection the DsRed expressing colonies and cells in each well were counted using a Nikon Eclipse TE200 fluorescence microscope. After 3 weeks, fresh growth-arrested feeder cells were added to each existing well or the spermatogonia were passaged into new wells containing fresh growth-arrested feeder cells. To passage the spermatogonia, loosely attached colonies were first removed from the well and dissociated with EDTA (0.25% EDTA in PBS) and then the remaining colonies were dissociated by trypsinization (0.25%, Invitrogen, 1 min). All of the dissociated spermatogonia were combined, washed in medium and re-plated. FGSC cultures were initiated and maintained as described in previous study [7].

### RNA Extraction and RT-PCR Analysis

Total RNA was prepared from tissues or cultured cells using Trizol reagent (Invitrogen) followed by DNase treatment (Ambion). The cDNA was synthesized using MMLV-RT (Promega) according to manufacturer’s instructions. The sequences of the primers used for RT-PCR analysis were: *bmp2a* (Fwd1∶5′- ACTTCGGCTTCTGAGCATGT -3′/Rev1∶5′- GTCCGTCTGTGGTCCACTTT -3′); *bmp2b* (Fwd2∶5′-CCAGCAGAGCAAACACGATA-3′/Rev2∶5′-GACCGTCATGGCTGTAGGTT-3′); *bmp4* (Fwd3∶5′-AGATCCACCAGTCGAGCCAA-3′/Rev3∶5′-TGCCGTCATGTCCGAATGTG-3′); *dazl* (Fwd4∶5′-GAAGCATCGTCAGGGTTT-3′/Rev4∶5′- GATGACACTGACCGAGAAC-3′); *dnd* (Fwd5∶5′- TCTGCAGGAATGGATGCAGAGGAA-3′/Rev5∶5′- TCTGACGGTGATGGAAATGCCGTA-3′); *nanos3* (Fwd6∶5′- AGCCTTGGAAGGACTACATGGGTT-3′/Rev6∶5′- TGATTTGGCGTACACCGAGCAGTA-3′); *vasa* (Fwd7∶5′-GCAGGACCCAAGGTTGTTTA-3′/Rev7∶5′- GCACTTTACTCAGGCCAATCT-3′); *piwil1* (Fwd8∶5′-CTCAGAGGTTTAGAACTACGTGAGGG-3′/Rev8∶5′- GTGGGATGTTGAATGGGTCATCAGGA-3′); *β-actin* (Fwd9∶5′-AGACATCAGGGTGTCATGGTTGGT-3′/Rev9∶5′-TGGTCTCGTGGATACCGCAAGATT-3′); *plzf* (Fwd10∶5′-TGCCACGCTCCAAGCTAAAGTAGA -3′/Rev10∶5′-TTCCTGTGTTGCTCTATGGCCTCA -3′); *sox17* (Fwd11∶5′-AAACGAAACAAGCGATTGGAGCCC-3′/Rev11∶5′-TGACCAGAACTGTGGGTTGCTGTA-3′). The PCR program was 94°C (1 min), 35 cycles at 94°C (10 sec)/55°C (10 sec)/68°C (1 min).

### Cell Transplantation and Analysis

Cultured spermatogonia were dissociated (0.25% EDTA in PBS), washed, re-suspended in 50 µl of L-15 medium and immediately transplanted into two-week-old recipient larvae that were treated as embryos with a morpholino (MO) nucleotides against *dnd* [23]. Cell transplantations were performed under a stereomicroscope using a glass micropipette needle. Spermatogonia were transplanted into the abdominal cavity under the swim bladder close to the gonads according to a published method [19]. Two weeks after transplantation, the recipients were examined by fluorescence microscopy and the potential germline chimeras were identified based on the presence of DsRed-positive cells in the gonadal region. To determine if the transplanted cells were able to generate functional gametes, the recipient fish were raised to sexual maturity and paired with wild-type zebrafish mates.

### Statistical Analysis

Data obtained from the growth assays were presented as the mean and standard deviation. For statistical analysis Student t-tests or one-way ANOVA was applied followed by Bonferroni-Dunn tests using SAS program. The significance was accepted at *p<*0.05.

## Results

### Derivation of Spermatogonial Cell Cultures from *Tg(piwil1:neo);Tg(piwil1:DsRed)* Zebrafish

Immunocytochemical analysis of testicular tissue dissected from *Tg(piwil1:neo)* fish confirmed that Neo expression overlapped with Vasa in the spermatogonial cells (Fig. 1A–C) indicating that a drug selection approach could be used to isolate the germ cells in culture. To initiate spermatogonial cell cultures, an enriched fraction of DsRed-positive testicular germ cells was obtained by Percoll separation of dissociated testes dissected from *Tg(piwil1:neo);Tg(piwil1:DsRed)* fish. The germ cell fraction was seeded onto confluent growth-arrested OFC3 feeder cells that were engineered to express zebrafish Lif and Fgf2 (OFC3LF) or Lif and Gdnf (OFC3LG) [7] and G418 was added to eliminate any remaining somatic cells. Following 3 weeks of drug selection colonies of 4 or more DsRed-positive spermatogonia were observed in the culture (Fig. 2A–D). The small (about 10 µm-diameter) DsRed-positive cells possessed morphological characteristics of spermatogonia in the testis [19] with round nucleus and a high nucleus-to-cytoplasm ratio (Fig. 2A,B). Cell counts performed on 3 week-old cultures revealed that the number of DsRed-positive, G418-resistant spermatogonia was significantly greater on OFC3LF and OFC3LG feeder layers compared to the parent OFC3 feeder line (Fig. 2E). After 3 weeks the cell number began to dramatically decrease in all of the cultures resulting in only 5–10% of the cells remaining in cultures maintained for 6 weeks on OFC3LF and OFC3LG feeder layers (Fig. 2E).

**Figure 1:** Neo expression overlaps with Vasa in the testicular germ cells of *Tg(piwil1:neo)* fish. Photomicrographs showing that (A) Neo (green) and (B) Vasa (red) are expressed in the same testicular germ cells including the spermatogonia of *Tg(piwil1:neo)*; (C) merged photo of A and B. The section was also stained with DAPI (Blue). Scale bar = 20 µm.

**Figure 2:** Feeder cells expressing zebrafish Lif, Fgf2 and Gdnf promote spermatogonial cell proliferation for 3 weeks in culture. Photomicrographs showing G418-selected spermatogonia that were initiated from *Tg(piwil1:neo);Tg(piwil1:DsRed)* zebrafish showing (A) 4-cell and (B) 15-cell colonies; DsRed expression in the (C) 4-cell and (D) 15-cell colonies. (E) OFC3LF and OFC3LG significantly enhanced spermatogonial cell proliferation in cultures maintained for 3 weeks while the mitogenic effect was lost after 6 weeks. * indicates a significant difference by Student t-tests. Scale bar = 20 µm.

### Addition of Dorsomorphin Prolonged Spermatogonial Cell Growth but Inhibited FGSC Survival in Culture

The decrease in cell number observed in the spermatogonial cell cultures after 3 weeks was most likely due to differentiation of the spermatogonia since the DsRed-expressing cells became smaller and formed aggregates that detached from the feeder layer as described in previous studies of zebrafish spermatogonial cell cultures [13]. Analysis of the feeder cells by RT-PCR revealed that *bmp2a*, *bmp2b* and *bmp4* were all expressed by the OFC3LF and OFC3LG cells (Fig. 3A) raising the possibility that Bmp signaling may be involved in inducing spermatogonial differentiation. To test this hypothesis, spermatogonial cell cultures were initiated and maintained in the presence of dorsomorphin, an inhibitor of the Bmp type I receptor. Results from growth assays revealed that the addition of dorsomorphin significantly enhanced the proliferation of spermatogonia in 3 week-old cultures (Fig. 3B) with the greatest mitogenic effect observed when the inhibitor was added at a concentration of 2 µM. At this concentration of dorsomorphin, the growth rate of DsRed-expressing spermatogonia increased 80% compared to the control with several large colonies containing more than 60 cells present in the cultures (Fig. 3C). In 6 week-old cultures the presence of dorsomorphin increased the number of spermatogonia by 30-fold compared to the control (Fig. 4A) and DsRed-positive colonies containing more than 100 cells were observed (Fig. 4B). Results of RT-PCR analysis demonstrated that cultured spermatogonia continued to express the germ-cell markers *dazl*, *dnd, nanos3*, *vasa* and *piwil1* and the spermatogonial markers *plzf* and *sox17* [24], [25] for at least 6 weeks in the presence of dorsomorphin (Fig. 4C). In contrast, when dorsomorphin was added to drug-selected FGSC cultures [7] cell growth was significantly inhibited compared to controls maintained in the absence of dorsomorphin (Fig. 5A–D). Also, the expression of germ cell markers was significantly reduced or completely lost by 3 weeks in the dorsomorphin-treated FGSC cultures (Fig. 5E).

**Figure 3:** Dorsomorphin promotes the growth of spermatogonia in 3 week cultures. (A) RT-PCR results showing that feeder cells (OFC3LF+OFC3LG) express *bmp2a*, *bmp2b* and *bmp4*. (B) Addition of dorsomorphin significantly (p<0.001) enhanced spermatogonial cell proliferation in 3 week cultures. (C) Merged bright field and UV photomicrographs showing a colony containing approximately 65 DsRed-expressing spermatogonia. Data points not sharing a letter (A, B, C) are significantly different by Bonferroni–Dunn tests. Scale bar = 20 µm.

**Figure 4:** Dorsomorphin increased the growth of spermatogonia in 6 week cultures. (A) Addition of dorsomorphin significantly (p<0.001) increased the growth of spermatogonia maintained in culture for 6 weeks. (B) Merged bright field and UV photomicrographs showing a colony containing more than 100 DsRed-expressing spermatogonia. (C) RT-PCR analysis of RNA isolated from spermatogonia maintained for 6-weeks in culture in the presence of dorsomorphin, whole testis tissue and feeder cells alone showing expression of germ cell specific marker genes, *dazl*, *dnd*, *nanos3*, *vasa* and *piwil1* and spermatogonial markers *plzf* and *sox17.* RT: reverse transcription; Data points not sharing a letter (A, B, C, D) are significantly different by Bonferroni–Dunn tests. Scale bar = 20 µm.

**Figure 5:** Dorsomorphin inhibits the growth of FGSCs in 3 week cultures. (A) Addition of dorsomorphin significantly inhibits FGSC (A) colony formation and (B) cell proliferation in culture. Photomicrographs showing (C) a 3-week old FGSCs (arrows) cultured in the presence of 2 µM dorsomorphin and (D) a 3-week-old FGSC colony cultured in the absence of dorsomorphin. (E) RT-PCR analysis of RNA isolated from a 3-week FGSC culture grown in the presence or absence of dorsomorphin, whole ovaries and feeder cells alone. Dorsomorphin severely reduced the expression of germ cell specific marker genes, *dazl*, *dnd*, *nanos3*, *vasa* and *piwil1*. * indicates a significant difference by Student t-tests. Scale bar = 20 µm.

### Dorsomorphin Enhanced the Capacity of Spermatogonial Cell Cultures to Colonize the Gonads and Produce Functional Gametes Following Transplantation to Recipient Fish

Cell transplantation experiments were performed to evaluate the germline competency of the spermatogonial cell cultures. Spermatogonia obtained from 3- or 6-week-old cultures were transplanted into recipient larvae that were treated as embryos with a MO nucleotides against *dnd* to block endogenous germ cell formation [23]. For each experiment approximately 20 to 60 spermatogonia were transplanted into the recipient larva. Due to the small number of cells available, only approximately 10 or less DsRed-expressing cells were transplanted in experiments involving spermatogonia cultured for 6 weeks in the absence of dorsomorphin. Two weeks after transplantation, the recipients were screened by fluorescence microscopy to identify those that possessed DsRed-positive cells in the gonadal region (Fig. 6A). Survivors were raised to sexual maturity and successful germline transmission of the transplanted cells was confirmed by pairing the chimeric fish with wild-type zebrafish mates. All of the surviving adult recipient fish that were obtained from the transplantation experiments were male. A total of 36 recipient male fish were obtained from 2 independent cell transplantations using 3 week-old spermatogonia cultured in the absence of dorsomorphin. Five of the fish (13.8%) were fertile and generated normal offspring (Table 1). When spermatogonia that were cultured for 3 weeks in the presence of dorsomorphin were transplanted, 10 of the 52 (19.2%) adult recipients obtained were fertile (Table 2). The presence of dorsomorphin had a dramatic effect on promoting the germline competency of 6 week spermatogonial cell cultures. None of the 28 adult recipients obtained by transplanting 6-week-old spermatogonia cultured without dorsomorphin were fertile while 9 of 50 (18%) recipients (Table 3) produced from the 6 week dorsomorphin-treated spermatogonia were able to reproduce. Genomic PCR analysis revealed 100% inheritance of *piwil1-neo* confirming that all of the offspring were derived from the transplanted spermatogonia (Fig. 6B). All of the fertile recipient fish obtained were able to produce multiple batches of normal offspring for at least 6 months. Dissection of three fertile recipients that were produced from transplanted 6-week-old spermatogonial cell cultures revealed that two of the fish developed only a single testis on one side of the body and the third fish developed two testes of unequal size (Fig. 6C). All of the testes examined contained DsRed-positive cells (Fig. 6C1). Histological examination of the fully-developed testes revealed the presence of a significant number of mature sperm along with spermatogonial cells at different developmental stages present in individual tissue sections (Fig. 6D). Results from cell transplantation experiments demonstrated the presence of SSCs in the spermatogonial cell cultures derived from the testes of *Tg(piwil1:neo);Tg(piwil1:DsRed)* zebrafish.

**Figure 6:** Germline transmission of spermatogonia cultured for 6 weeks in the presence of dorsomorphin. (A) Photomicrograph showing the incorporation of DsRed-positive cultured spermatogonia (arrow) into the gonad of a recipient larva two weeks after transplantation. (B) Results of genomic PCR showing the presence of *piwil1-neo* sequences that were inherited by all of the F1 individuals (lanes 1 to 16) produced by a germline chimeric father. Negative control: genomic DNA template from a wild-type larva (lane 17); positive control: pPiwil1-neo plasmid DNA template (lane 18). (C) Dissection of a fertile adult male recipient fish showing that the transplanted DsRed-positive spermatogonia have proliferated and directed the formation of a pair of unequal sized testes (arrow) in the body. (C1) Inset shows the gonad under UV light revealing the presence of DsRed-positive cells. (D) Transverse section of testis from a fertile recipient fish showing active spermatogenesis. Sb: swim bladder; S: spermatozoa (arrow). Scale bar = 100 µm for A and 20 µm for D.

**Table 1:** Results from two transplantation (T) experiments using 3-week-old spermatogonia cultured without dorsomorphin.

Exp. groups	Number of recipients transplanted	Number of recipients that survived to adulthood	Number and (%) of recipients carrying germline transmitted spermatogonial cells
T1	24	17	3 (18%)
T2	31	19	2 (11%)
Total	55	36	5 (14%)

**Table 2:** Results from three transplantation (T) experiments using 3-week-old spermatogonia cultured with dorsomorphin.

Exp. groups	Number of recipients transplanted	Number of recipients that survived to adulthood	Number and (%) of recipients carrying germline transmitted spermatogonial cells
T1	25	19	4 (21%)
T2	19	15	3 (20%)
T3	28	18	3 (17%)
Total	72	52	10 (19%)

**Table 3:** Results from three transplantation (T) experiments using 6-week-old spermatogonia cultured with dorsomorphin.

Exp. groups	Number of recipients transplanted	Number of recipients that survived to adulthood	Number and (%) of recipients carrying germline transmitted spermatogonial cells
T1	21	14	2 (14%)
T2	26	17	3 (18%)
T3	30	19	4 (21%)
Total	77	50	9 (18%)

## Discussion

In adult mammals, the SSC population in the testis is represented by the type A undifferentiated (A_und_) spermatogonia that are present as single (A_s_), paired (A_pr_) or multiple aligned (A_al_) cells [26], [27]. The type A_pr_ and A_al_ spermatogonia are able to dissociate to generate type A_s_ cells [28]. In contrast, the zebrafish testis possesses two subtypes of undifferentiated type A spermatogonia, A_und_ and A_und*_, that possess stem cell characteristics based on cell transplantation experiments [29], [30]. In this study we showed that Neo is expressed in the spermatogonia of the *Tg(piwil1:neo)* fish enabling us to use a drug selection approach to derive spermatogonial cell cultures initiated from the testes of *Tg(piwil1:neo);Tg(piwil1:DsRed)* fish. Using G418 selection to eliminate the somatic cells that were present in the testicular primary cultures enabled us to avoid the problem of the spermatogonia becoming overgrown in culture which was encountered in previous studies [13], [31]. Another advantage of using the *Tg(piwil1:neo);Tg(piwil1:DsRed)* fish was that the expression of *piwil1:DsRed* made it possible to visually evaluate the growth of the spermatogonia in culture by fluorescence microscopy. The zebrafish spermatogonial cell cultures were derived in conditions that were similar to those previously used to propagate zebrafish FGSCs in culture [7]. A unique requirement of the spermatogonial cell culture system, however, was to block Bmp signaling by the addition of dorsomorphin to the medium. Previous studies have shown that Bmp functions to promote spermatogonial differentiation both in vivo and in spermatogonial cultures. Mutation of the zebrafish Bmp type I receptor resulted in an impairment of spermatogonial differentiation in vivo while addition of BMP4 to mouse SSC cultures promoted the production of differentiated spermatids [14], [15], [16]. Since our analysis of the OFC3 feeder cells, used to derive our spermatogonial cell cultures, showed that the cells expressed *bmp2a, bmp2b and bmp4*, we decided to block Bmp signaling by adding dorsomorphin to the culture medium. Dorsomorphin, also known as compound C, is a small molecular weight inhibitor of the Bmp type I receptor [32]. The compound has been shown to disrupt dorsoventral patterning when it is administered to zebrafish embryos [33]. We found that in cultures maintained for 3 weeks in the absence of dorsomorphin the zebrafish spermatogonia became smaller and formed aggregates that detached from the feeder cells indicating that the cells had differentiated to non-proliferating spermatids [11]. Addition of dorsomorphin to the cultures inhibited differentiation and enabled the spermatogonia to proliferate and express appropriate markers for more than 6 weeks in vitro. Further evidence that dorsomorphin maintained the SSC characteristics in culture was obtained from the cell transplantation experiments showing that the presence of dorsomorphin extended the time that the cultured SSCs could be transplanted and colonize the gonads of recipient larvae and produce functional gametes in the adult chimeric fish. In contrast, when dorsomorphin was added to zebrafish FGSC cultures, the cells stopped proliferating and lost expression of the germ cell markers within 3 weeks, demonstrating a requirement for Bmp signaling by the female germ cells in culture. These results showing that Bmp signaling has the opposite effect on zebrafish male and female germline stem cells in culture may be useful in optimizing conditions that support the growth of germline stem cells from other species.

The OFC3 feeder cell line used to initiate the spermatogonial cell cultures was derived from ovaries obtained from *Tg(gsdf:neo)* zebrafish [7]. Gsdf is produced in somatic cells of the fish ovary and testis and functions to promote the growth of germ cells [34]. To derive OFC3, G418 selection was applied to *Tg(gsdf:neo)* ovarian primary cultures to isolate the Gsdf-expressing cells. Since OFC3 cells express Gsdf, it was expected that they may also produce other unknown factors that promote the growth and survival of germ cells in culture and therefore serve as an ideal feeder layer for spermatogonia. To optimize the spermatogonial cell culture conditions, OFC3 was transfected to express zebrafish Lif and Fgf2 (OFC3LF) or Gdnf (OFC3LG). Recombinant LIF, FGF2 and GDNF have all been shown to be important factors in establishing mouse SSC cultures [22], [35]. Previously, we demonstrated that optimal growth of zebrafish FGSCs was achieved using the OFC3LF and OFC3LG feeder layers indicating that the cells produce factors that support zebrafish germ cells in culture [7]. A previously reported zebrafish spermatogonial cell culture system employed a feeder cell line that was derived from a spontaneously arising zebrafish testicular tumor [11]. Although we made several attempts to establish a continuously-growing G418 resistant feeder cell line initiated from healthy *Tg(gsdf:neo)* testicular tissue, we were not successful.

Using the drug selection strategy and culture conditions that were developed in this study, spermatogonia could be propagated for several weeks in vitro and then transplanted into infertile recipient larvae where the cells colonized the gonads and generated fertile adult fish at a high frequency. Since recipient larvae were treated as embryos with a MO that blocked endogenous germ cell formation and gonad development resulting exclusively in the production of infertile male [23], the transplanted spermatogonia were able to direct the formation of a functional gonad and rescue fertility of the host fish. Although only approximately 60 spermatogonia were transplanted into each recipient, the fertile adult fish that resulted from the transplantations were able to produce multiple batches of offspring over a 6 month period. These results demonstrate that the transplanted cells re-established the entire spermatogonial cell lineage in the host testis and therefore possessed germline stem cell qualities that are characteristics of SSCs. Only male fertile recipients were produced from successful germline transmission of transplanted spermatogonial cells. Using germ cell ablation, a recent zebrafish study has suggested that signals from female germ cells, particularly the oocytes, may be needed to promote primary female sex determination and maintain female development throughout adulthood [36]. It is most likely that the cultured spermatogonial cells did not produce these signals that are required for female development. As such, all the fertile recipients completely developed into males. The spermatogonial culture system described in this study will provide an in vitro model for studies of extracellular factors controlling zebrafish spermatogonial differentiation and may form the basis of gene transfer approach.
